# Inhibition of Hepatitis C Virus Infection by DNA Aptamer against NS2 Protein

**DOI:** 10.1371/journal.pone.0090333

**Published:** 2014-02-28

**Authors:** Yimin Gao, Xiaoyan Yu, Binbin Xue, Fei Zhou, Xiaohong Wang, Darong Yang, Nianli Liu, Li Xu, Xiaohong Fang, Haizhen Zhu

**Affiliations:** 1 Department of Molecular Medicine, State Key Laboratory of Chemo/Biosensing and Chemometrics, Hunan University, Changsha, China; 2 Research Center of Cancer Prevention & Treatment and Translational Medicine Research Center of Liver Cancer, Hunan Provincial Tumor Hospital (Affiliated Tumor Hospital of Xiangya Medical School of Central South University), Changsha, China; 3 Key Laboratory of Molecular Nanostructure and Nanotechnology, Institute of Chemistry, Chinese Academy of Sciences, Beijing, China; Academia Sinica & National Defense Medical Center, Taiwan

## Abstract

NS2 protein is essential for hepatitis C virus (HCV) replication. NS2 protein was expressed and purified. Aptamers against NS2 protein were raised and antiviral effects of the aptamers were examined. The molecular mechanism through which the aptamers exert their anti-HCV activity was investigated. The data showed that aptamer NS2-3 inhibited HCV RNA replication in replicon cell line and infectious HCV cell culture system. NS2-3 and another aptamer NS2-2 were demonstrated to inhibit infectious virus production without cytotoxicity in vitro. They did not affect hepatitis B virus replication. Interferon beta (IFN-β) and interferon-stimulated genes (ISGs) were not induced by the aptamers in HCV-infected hepatocytes. Furthermore, our study showed that N-terminal region of NS2 protein is involved in the inhibition of HCV infection by NS2-2. I861T within NS2 is the major resistance mutation identified. Aptamer NS2-2 disrupts the interaction of NS2 with NS5A protein. The data suggest that NS2-2 aptamer against NS2 protein exerts its antiviral effects through binding to the N-terminal of NS2 and disrupting the interaction of NS2 with NS5A protein. NS2-specific aptamer is the first NS2 inhibitor and can be used to understand the mechanisms of virus replication and assembly. It may be served as attractive candidates for inclusion in the future HCV direct-acting antiviral combination therapies.

## Introduction

Hepatitis C virus (HCV) infects approximately 3% of the world population, leading to chronic hepatitis, liver cirrhosis and even hepatocellular carcinoma [1]. Peginterferon alpha-based therapy is efficacious in part of the selected individuals and associated with side effects [2]. The protease inhibitors against NS34A have been recently approved by US FDA for patients infected with HCV genotype 1. However, mutant viruses resistant against these drugs have emerged in vitro and in vivo, suggesting that several enzymatic activities or viral functions may have to be targeted in parallel in a combination approach, similar to the highly active antiretroviral therapy (HAART) against human immunodeficiency virus [3].

HCV is a small enveloped virus belonging to the *Hepacivirus* genus in the *Flaviviridae* family. It possesses a single positive-strand RNA genome encoding a long polyprotein which is processed by cellular and viral proteases into 10 different proteins, including structural proteins (core, E1, and E2) and non-structural proteins (p7, NS2, NS3, NS4A, NS4B, NS5A, and NS5B). NS2 contains several putative transmembrane segments in the N-terminal region and a carboxy-terminal cytoplasmic region. The C-terminal domain (residues 94–217) of NS2, together with residues 1–181 of NS3, forms the NS2/3 protease. Dimerization of NS2/3 was required for proteolytic activity and therefore initiation of the viral RNA replication [4], [5]. NS2 protein has been shown to be required for infectious virus production [6]–[8]. The essential role of NS2 in HCV lifecycle makes it an attractive target for antiviral therapies. The development of in vitro infectious HCV culture systems derived from genotype 2a (JFH1) and genotype 1a (H77S) has facilitated the study of HCV lifecycle and provides powerful tools for the discovery of novel antiviral drugs [9]–[12].

Aptamers are artificial nucleic acid ligands that bind to their targets with high affinity and specificity. They can be obtained by the selective evolution of ligands by exponential enrichment approach (SELEX) in vitro [13], [14]. SELEX involves a series of enrichment cycles and counter selection based on repetitive binding that ultimately selects for a group of aptamers binding to the targets. Aptamers can specifically recognize the targets or regulate their functions. Aptamers have numerous advantages over antibodies because of their high specificity to their targets, convenient synthesis, no immunogenicity, and long-term stability [15], [16].

Here we obtained the aptamers for NS2 protein using SELEX. The data demonstrated that NS2-2 aptamer against NS2 protein exerts its antiviral effects through binding to the N-terminal of NS2 and disrupting the interaction of NS2 with NS5A protein.

## Materials and methods

### Cells, plasmids and reagents

FL-Neo, a HCV 1b full-length replicon cell line, Huh7.5 cells, pFL-JC1 (chimera containing a J6-JFH1 junction between the first and second putative transmembrane domains of NS2) and mouse monoclonal anti-NS2 antibody (6H6) were kindly provided by Charles Rice (Rockefeller University, New York, NY) [10], [17]. pJFH1 and pJFH1/GND plasmids were generously provided by Takaji Wakita (National Institute of Infectious Diseases, Tokyo, Japan) [11]. pH77S and pH77-S/ΔE1P7 were obtained from Stanley Lemon (University of North Carolina, Chapel Hill, NC) [9]. Mouse monoclonal anti-NS5A antibody was a gift from Chen Liu (University of Florida, Gainesville, FL).

### Expression and purification of HCV NS2 protein

The entire NS2 was PCR amplified from plasmid pJFH1, digested with NdeI and EcoRI, and inserted into pET-28b(+) (Novagen, Madison, MI) to produce pET28b-NS2 construct. NS2 protein was expressed in *Escherichia coli* BL21 cells (Invitrogen, Carlsbad, CA). The NS2 protein was purified and identified using anti-His antibody (Sigma, St Louis, MO) via western blot described below.

### In vitro selection of aptamers against HCV NS2

The synthesized DNA library pool with an overall complexity of ∼10^14^ was used for in vitro selection. The sequence of the random DNA is 5′-ACGCTCGGATGCC ACTACAG(N40)CTCATGGACGTGCTGGTGAC-3′, where N40 represents 40 nucleotides with equal molar incorporation of A, G, C, and T at each position. The selection and amplification procedure was performed as previously described [16], [18]. After 6 rounds of selection, the amplified DNA was cloned and several clones were sequenced.

### Enzyme-linked oligonucleotide assay (ELONA)

Streptavidin-precoated microtiter plates were coated with biotin-labeled aptamer. The plates were washed thrice with PBS containing 1 mM MgCl_2_, 0.1% BSA, 0.05% Tween-20. Serial dilutions of His-tagged NS2 protein was added into the plates and incubated at 37°C for 30 min. After washing to remove the unbound target protein, mouse against His or NS2 monoclonal antibody was added into the plates. After incubation at 37°C for 1 hour, horseradish peroxidase-labeled goat anti-mouse IgG was added and incubated at 37°C for 30 minutes. Color development was performed by addition of freshly prepared substrate solution for 10 min at room temperature. After stopping the reaction with stopping buffer, the plates were read with ELISA reader and the absorbance of each sample was measured at 450 nm.

### Generation of plasmids expressing different truncated versions of NS2

Different truncated versions of NS2 were amplified from pJFH1 using the following primers and cloned into the expression vector pcDNA3.1/V5-His (Invitrogen, Carlsbad, CA). NS2-F1 forward 5′-CTGCAGTCTAGAGCAGAATATAGTGACGG -3′ and reverse 5′-CTGCAGTCTAGACTAGTCTCCGCCGTGAT-3′ are for NS2-F1. NS2-F2 forward 5′-CGCGCGGATCCATGTATAAGACCCTCCTC-3′ and reverse 5′-CTGCAGTCTAGATAAGAGGTAAGCAGGCC-3′ are for NS2-F2. NS2-F3 forward 5′-CGCGCGGATCCATGAGGGCCGCTTTGACA-3′ and reverse 5′-CTG CAGTCTAGAAAGGAGCTTCCACC -3′ are for NS2-F3.

### MTS assay

The procedure was previously described [18]. Briefly, one day before treatment, 1.0×10^3^ cells were seeded in triplicate in a 96-well plate. The cells were cultured with or without aptamer for indicated time periods at 37°C. Twenty microliter of the CellTiter AQ Solution containing MTS and an electron coupling reagent (Promega) was added to each well. After 2 hours incubation at 37°C, the absorbance at 490 nm was measured. Cell viability was calculated with respect to the control samples. Three independent experiments were performed in triplicate.

### Real-time PCR assays

Aptamer or library was delivered into viral-infected cells by transfection with lipofectamine 2000 for different time periods. Total cellular RNA was isolated using TRIzol (Invitrogen, Carlsbad, CA). The primers targeted HCV, HBV, GAPDH, IFN-β, G1P3 and 1-8U have been reported and real-time PCR was performed as published previously [19].

#### Selection of resistance-conferring mutations

HCV-infected Huh7.5 cells were treated with 100 nM NS2-2 for 2 weeks. Control cells were maintained with 100 nM library. NS2 cDNA was recovered from cells by RT-PCR. NS2 amplicons were used for direct population sequencing and to generate cDNA clones with a TOPO-TA cloning kit (Invitrogen). The substitution I861T was introduced into pJFH1 plasmid by using QuickChange site-mutagenesis kit (Stratagene). In vitro transcripts of wild type JFH1 and selected mutated I861T JFH1 were generated and transfected into Huh7.5 cells respectively.

### Western blot analysis

The procedure was previously described [20]. Briefly, cells were washed with PBS and lysed in RIPA buffer. Twenty micrograms of protein were resolved by SDS/PAGE, transferred to a PVDF membrane and probed with appropriate primary and secondary antibodies. The bound antibodies were detected by ECL reagent (Pierce, Rockford, IL) according to the manufacturer's instruction.

#### Co-Immunoprecipitation (IP) and immunoblotting

HCV-infected Huh7.5 cells in 60 mm culture dish were washed thrice with ice-cold PBS containing 0.25 M glycine. The cells were lysed in 100 µL of lysis buffer (25 mM Tris-HCl [pH 7.4] containing 150 mM NaCl, 1% NP-40, 1 mM EDTA and 5% glycerol) supplemented with protease inhibitors cocktail and incubated for 5 min at 4°C. Cell lysates were incubated for 30 min at 4°C, and centrifuged at 12,000 g for 15 min at 4°C. Dilute the lysate before beginning IP to 2 µg/µl total cellular protein with PBS. Two hundred micrograms of lysates were immunoprecipitated with 15 µl of anti-NS5A antibody by gently rocking the reaction mixture at 4°C overnight. Capture the immunocomplex by adding 30 µl of washed Protein G Agarose bead slurry and gently rock the reaction mixture at 4°C for 4 hours. Wash the beads 3 times with PBS. The proteins binding to the beads were boiled in 60 µl of 2×Laemmli sample buffer and then subjected to SDS–12% PAGE for immunoblot.

### Intracellular virus preparation

At the indicated time postinfection, cells were washed thrice with PBS and incubated with 0.25% of trypsin-EDTA (Invitrogen, Carlsbad, CA) for 2 minutes at 37°C. Cells were suspended in PBS and collected by centrifugation at 2000 rpm for 3 minutes. The cell pellet was resuspended in DMEM, and lysed by four freeze-thaw cycles at liquid nitrogen and 37°C water bath, respectively. Cell debris was pelleted by centrifugation for 5 minutes at 4000 rpm. The supernatant was collected and used for focus-forming units assay described below.

### Focus-forming units (FFU) assay

The protocol was performed as previously reported [12]. Briefly, cell supernatants were serially diluted 10-fold in complete DMEM and used to infect 10^4^ naïve Huh7.5 cells per well in 96-well plates. The inoculums were incubated with cells for 1 hour at 37°C and then supplemented with fresh DMEM. The level of HCV infection was determined 3 days postinfection by immunofluorescence staining for NS5A. The viral titer is expressed as focus-forming units per milliliter of supernatant (FFU/mL), determined by the average number of NS5A-positive foci detected at the highest dilutions.

### Statistical analysis

Differences between means of reading were compared using Student *t*-test. Error bars represented S.D.

## Results

### Purification of HCV NS2 protein and selection of aptamers against NS2 protein

To generate aptamers for HCV NS2, the cDNA fragment encoding the NS2 gene of JFH1 was amplified by PCR. The amplified product was cloned into the expression vector pET-28b(+) and confirmed by DNA sequencing. NS2 protein was expressed and purified by its N-terminal His-tag. The purified NS2 protein was confirmed by western blot and Coomassie Brilliant Blue staining (Figure 1A).

**Figure 1:** Binding of DNA pools from round 1 and round 6 to NS2 protein. (**A**) Western blot analysis of purified NS2 protein. His-tagged NS2 was expressed by IPTG induction in *E. coli* BL21 and then confirmed using mouse anti-His monoclonal antibody via western blot (left) and Coomassie Brilliant Blue staining (right). (**B**) Comparison of fluorescence of different pools of FITC-labeled DNA binding to NS2 protein or control LacZ protein. FITC-labeled DNA pools from round 1 or round 6 were incubated with nickel beads conjugated with NS2 or control protein. The density of the fluorescence was measured and normalized to library. Results are the average of three independent experiments. ^**^ *P*<0.01 verse library.

A nucleotide library was obtained from a pool of ∼10^14^ single-stranded DNA molecules containing a random segment of 40 nucleotides flanked by 5′ and 3′ constant primers as conserved linkers to amplify the selection process. The DNA pool was mixed with His-tagged NS2 protein. DNA-NS2 protein complexes were precipitated with nickel beads, and pellets were washed. DNAs were recovered, amplified with PCR, and used for next rounds of selection. Six subsequent rounds of selection were performed. There was a marked increase in the binding of round 6 DNA pools to NS2 protein compared to that of the pools of round 1 (Figure 1B). The selected aptamers were cloned and sequenced. A total of 104 clones from the DNA pools of round 6 were sequenced. The topmost sequence was used as a representative member for the study. The aptamers were named NS2-1, NS2-2 and NS2-3 respectively. The sequences of these aptamers are CTGGATCGA AAAGTATCCACGTTTGTCTGAAAATAGTGGCC, CAGGTACCACCTTCATGG GCGCGGAAGACGATGGTGTACTA, ACGGGGCAGGATTGTCCCCGCGCCTG GTTGAAGGTAGTCGC respectively.

### Analysis of binding affinity of NS2-specific aptamers

To determine the binding affinity of individual aptamer to NS2 protein, ELONA assay was performed with each aptamer and NS2 protein. Aptamers NS2-1, NS2-2 and NS2-3 showed high affinity for recombinant NS2 protein compared with the library (Figure 2A). Various aptamers bound to NS2 protein and this interaction was retained even in the presence of excess yeast tRNA, indicating that their binding to NS2 was specific. We tested whether the aptamers NS2-1, NS2-2 and NS2-3 could bind NS2 protein in the lysates of HCV-infected hepatocytes. As shown in Figure 2B, aptamers against NS2 showed higher binding affinity to NS2 protein in the lysates of viral infected cells compared with the library while they displayed no apparent binding affinity to core or NS5A protein in the lysates viral infected cells. Core, NS2 or NS5A protein in the lysates of HCV-infected Huh7.5 cells could be detected by antibodies against HCV core, NS2 or NS5A respectively (Figure 2B, lower panel). Co-localization of NS2-specific aptamers with NS2 protein in the HCV-infected hepatocytes was demonstrated in Figure 2C.

**Figure 2:** Binding affinity of selected aptamers against NS2. (**A**) The binding affinity of aptamers NS2-1, NS2-2 or NS2-3 to recombinant NS2 protein. Biotin-labeled each aptamer was added to the microtiter plate previously coated with streptavidin. Purified NS2 protein or control LacZ protein was added to the plates. ELONA assay was performed. The absorbance was normalized to the library and represented means of 3 different experiments performed in triplicate. ^**^ *P*<0.01 verse library. (**B**) The binding affinity of aptamers against NS2 to NS2 protein in the lysates of HCV-infected Huh7.5 cells. The plates were treated as described in part A. Lysates of HCV-infected Huh7.5 cells or control Huh7.5 cells were added to the plates. Mouse anti-NS2, anti-core or anti-NS5A monoclonal antibody was used. The absorbance was normalized to the library and represented means of three independent experiments performed in triplicate (upper). ^*^ *P*<0.05, ^**^ *P*<0.01 verse library. Core, NS2 or NS5A protein in the lysates of HCV-infected Huh7.5 cells and naïve Huh7.5 cells was detected by western blot using antibodies against HCV core, NS2 or NS5A respectively (lower). (**C**) Co-localization of NS2-specific aptamers with NS2 protein in the HCV-infected hepatocytes. HCV-infected Huh7.5 cells were treated with Cy5-labeled aptamers for 24 hours. The cells were fixed with ice-cold acetone for 10 minutes at −20°C. The cells were washed with PBS, blocked with 1:50 goat serum for 30 minutes at room temperature and then incubated for 1 hour with mouse monoclonal anti-NS2 antibody. The cells were stained with Texas Red-labeled goat anti-mouse for 45 minutes respectively at room temperature. The nuclei were counterstained with DAPI. Fluorescent images were obtained under fluorescent microscope. Identical setting was maintained for images capture. Representative images are shown.

### Inhibition of HCV infection by aptamers against NS2

To test whether NS2 aptamers inhibit HCV RNA replication, we treated full-length replicon cell line FL-neo with the aptamers. The level of HCV RNA was lower in NS2-3-treated cells than in library-treated group (Figure 3A). We decided to test whether NS2-specific aptamers inhibit HCV infection in infectious cell culture system. JFH1 virus suspension at multiplicity of infection (MOI) of 0.1 was used to infect Huh7.5 cells for 3 days and the viral-infected cells were treated by different doses of NS2-specific aptamers. The viral RNA was lower in NS2-3-treated cells than in library-treated group (Figure 3B). The concentration of aptamers used in the study showed no apparent toxic effect to the cells (Figure 3C).

**Figure 3:** Inhibition of HCV infection by aptamers against NS2. (**A/B**) Effect of NS2-specific aptamers on viral RNA replication in HCV full-length replicon cell (A) or HCV-infected Huh7.5 cells (B). FL-neo (A) or HCV-infected Huh7.5 cells (B) were treated with aptamer NS2-1, NS2-2 or NS2-3 for 72 hours. Intracellular HCV RNA was detected with real-time PCR and normalized with GAPDH. The data represented means of three different experiments. (**C**) The effect of NS2 aptamer on cell viability. HCV-infected Huh7.5 cells were treated by 100 nM or 200 nM aptamers for 72 hours. The effect of aptamer on cell viability was measured by MTS assay. The data were normalized with the control and represented means of three independent experiments performed in triplicate. (**D**) Titration of HCV particles produced in HCV-infected Huh7.5 cells with aptamer treatment by FFU assay. HCV-infected Huh7.5 cells were treated as described in part B. The cell culture supernatants and intracellular virus particles were harvested and titered by FFU assay. The infectivity titers in the supernatant or inside the cells are the average of three different experiments. (**E**) Effect of aptamers on H77-S viral RNA replication (upper) and the production of viral particles (lower) in infectious cell culture system. H77-S–infected Huh7.5 cells were treated with 100 nM of each aptamer or library for 72 hours. Intracellular viral RNA was quantified by real-time PCR and normalized with GAPDH. The data represented means of three independent experiments. The cell culture supernatants were harvested and titered by FFU assay. The infectivity titers in the supernatant are the average of three different experiments. (**F**) Effect of aptamers on JC1 viral RNA replication (upper) and the production of viral particles (lower). JC1 RNA was in vitro transcript from the plasmid pFL-JC1. JC1 RNA was transfected into Huh7.5 cells and JC1 virus was collected from the cells. JC1 virus was used to infect Huh7.5 cells in the presence of 100 nM aptamer for 72 hours. Intracellular viral RNA was quantified by real-time PCR and normalized with GAPDH. The data represented means of three independent experiments. The cell culture supernatants were harvested and titered by FFU assay. The infectivity titers in the supernatant are the average of three different experiments. (**G**) Effect of NS2-specific aptamers on hepatitis B viral DNA replication. HepG2.2.12 cells were inoculated with 100 nM of aptamer for 72 hours. Intracellular HBV DNA was detected with real-time PCR and normalized with GAPDH. The data represented means of three different experiments. ^*^ *P*<0.05, ^**^ *P*<0.01 verse library.

To examine whether aptamers against NS2 inhibit the production of viral particles, we harvested the supernatant of HCV-infected cells with aptamer treatment and used it to infect naïve Huh7.5 cells. The viral-infected Huh7.5 cells were revealed with anti-HCV NS5A antibody and numbered under a fluorescent microscope. The number of NS5A-positive foci (FFU) in Huh7.5 cells infected by secreted virus from viral-infected cells with NS2-3 treatment decreased in comparison with the control cells (Figure 3D). Interestingly, the level of extracellular infectious viruses was reduced 70% in the cells with NS2-2 treatment in comparison with library-treated cells (Figure 3D), although NS2-2 did not have marked effect on HCV RNA level (Figure 3B). We want to know whether the decrease in the extracellular infectious virions brought about by NS2-2 is due to defective virus assembly or impaired release of infectious virus particles. The level of intracellular infectious viruses was reduced 50% in the cells with NS2-2 treatment in comparison with library-treated cells (Figure 3D). These data suggested that aptamer NS2-2 inhibits both the virus assembly and release.

In addition, we examined the effect of the aptamer on HCV genotype 1a infection in human hepatocytes. H77-S RNA was in vitro transcript from the plasmid pH77-S. H77-S RNA was transfected into Huh7.5 cells and H77-S virus was collected from the cells according to the literature reported previously [21]. H77-S virus was used to infect Huh7.5 cells in the presence of aptamer. The viral RNA and the production of viral particles were reduced in aptamer-treated cells in comparison with the cells with library treatment (Figure 3E). Similarly, NS2-2 inhibited JC1 infection (Figure 3F). NS2-specific aptamers did not affect hepatitis B viral DNA replication (Figure 3G), implying that the aptamers against NS2 specifically inhibit HCV infection. All the data suggest that aptamers for NS2 inhibit HCV infection.

### NS2-specific aptamers do not trigger an innate immune response in viral-infected Huh7.5 cells

The presence of DNA molecules inside or outside the cells may trigger nonspecific innate immunity, which likely leads to antiviral effect. To exclude the possibility that the anti-HCV effect of NS2 aptamers is due to the aptamer-induced innate immunity, we tested the expression of IFN-β and IFN-stimulated genes (ISGs) in aptamer-treated cells. IFN-β was not induced in hepatocytes by aptamer treatment (Figure 4A). Our previous study demonstrated that G1P3 and 1-8U play an important role in the establishment of intracellular antiviral state [22]. We performed real-time PCR analysis to examine the expression of G1P3 and 1-8U in viral-infected cells with aptamers treatment. NS2-specific aptamers did not induce G1P3 and 1-8U (Figure 4B and 4C). All the data supported that inhibition of HCV infection by NS2-specific aptamers is not due to the innate immunity.

**Figure 4:** NS2-specific aptamers do not trigger innate immunity in HCV-infected Huh7.5 cells. HCV-infected Huh7.5 cells were treated by 100 nM aptamer or library for 24, 48 hours. Total cellular RNA was isolated. The level of IFN-β (**A**), G1P3 (**B**) and 18U (**C**) mRNA was quantified by real-time PCR and normalized with GAPDH respectively. IFN-a treatment was used as positive control. The data represented means of three different experiments. *P<0.05, **P<0.01, *** *P*<0.001 verse library.

### N-terminal region of NS2 protein is involved in the antiviral effects mediated by NS2-specific aptamer

To identify the residues of NS2 involved in aptamer binding and antiviral activity, we generated different truncated versions of NS2. The schematic of NS2 is shown in Figure 5A. The expression of different truncated versions of NS2 protein was verified (Figure 5B). ELONA assay was used to determine which truncated version binds to the aptamer NS2-2 and NS2-3. As shown in Figure 5C, transfection with the fragment I of NS2 (NS2-F1) (1–72 aa) or fragment III of NS2 (NS2-F3) (94–217 aa) had little affinity for aptamer NS2-2, whereas the fragment II of NS2 (NS2-F2) (26–93 aa) bided specifically to NS2-2. The data indicate that the binding region of aptamer NS2-2 localizes in the region between amino acid 26–93. The binding region of the aptamer NS2-3 localizes in the region between amino acid 1–72. To further verify that the aptamer NS2-2 binds to NS2-F2 and inhibits viral infection, we conducted competition experiments. NS2-F2 reversed the antiviral effects of the aptamer NS2-2 (Figure 5D). Taken together, the data suggested that the aptamer NS2-2 exerts its antiviral effects via interaction with NS2 in the region between aa 26–93.

**Figure 5:** N-terminal region of NS2 protein is involved in the antiviral effects of NS2-specific aptamer. (**A**) Schematic of NS2. (**B**) Confirmation of the expression of different truncated versions of NS2 protein. Different truncated versions of NS2 gene were amplified and cloned into pcDNA3.1/V5-His. Huh7.5 cells were transfected by these plasmids. Different truncated versions of NS2 protein were confirmed using anti-His antibody by western blot. (**C**) Binding affinity of different truncated versions of NS2 to the aptamer. The cells were treated as described in part B. The protein was isolated from the cells and binding affinity of truncated versions of NS2 to aptamer was determined by ELONA assay. The empty vector pcDNA3.1/V5-His was used as a control vector. The data represented means of three independent experiments performed in triplicate. *P<0.05 verse library. (**D**) Titration of HCV particles produced in HCV-infected cells transfected by truncated versions of NS2 with aptamer treatment. HCV-infected Huh7.5 cells were transfected by different truncated versions of NS2. Then the cells were treated by aptamer NS2-2 or library for 72 hours. The cell culture supernatants were harvested and titered by FFU assay on naïve Huh7.5 cells. The infectivity titers are the average of three independent experiments. *P<0.05 verse vector-transfected cells.

#### NS2-specific aptamer disrupts the interaction of NS2 with NS5A protein

Interaction of NS2 with NS5A protein is critical for infectious HCV production [6], [23]. Disruption the interaction of NS2 with NS5A protein may decrease infectious virus production. To address this hypothesis, we used immunoprecipitation to analyze the interaction of NS2 with NS5A protein directly. The amounts of NS2 or NS5A protein were comparable in aptamer or library-treated cells (Figure 6A). NS2 protein in the immunoprecipitates with equal amount of NS5A protein was lower in aptamer-treated cells than in library-treated group (Figure 6B). The data showed that NS2-2 blocked the interaction of NS2 with NS5A protein in HCV-infected hepatocytes. All the data suggested that NS2-specific aptamer NS2-2 inhibits HCV infection through blocking the interaction of NS2 with NS5A protein.

**Figure 6:** NS2-specific aptamer disrupts the interaction of NS2 with NS5A protein. (**A**) Protein was isolated from the HCV-infected Huh7.5 cells with aptamer or library treatment. The whole cell lysates (WCL) were used as input control. The input NS2 or NS5A protein was detected with western blot and quantified by densitometry. Results are the average of three independent experiments. (**B**) Effect of NS2-specific aptamers on the interaction of NS2 with NS5A protein. Protein was isolated from the HCV-infected Huh7.5 cells with aptamer or library treatment and immunoprecipitated with antibodies against NS5A or mouse IgG conjugated with agarose beads respectively. The protein binding to the beads were boiled and subjected to SDS-PAGE. The protein was transferred onto PVDF membrane and then reacted with mouse monoclonal anti-NS2 or NS5A antibody and secondary antibodies. NS2 protein was detected with western blot and quantified by densitometry in comparison with NS5A protein in the immunoprecipitates. *P<0.05, ** *P*<0.01 verse library-treated cells.

### Isolation and characterization of JFH1-resistant variants

Viral target-based inhibitor allows for the selection of resistant virus. To identify amino acid mutations that confer resistance to NS2 aptamer, HCV-infected Huh7.5 cells were treated with 100 nM NS2-2 for 2 weeks. Control cells were maintained with 100 nM library. Mutations within NS2 associated with reduced susceptibility to NS2-2 were selected and identified by sequence analysis of NS2 cDNA from control and aptamer-treated cells. Substitution at NS2 residue 861 (I861T substitution) was identified.

To evaluate the contribution of the selected specific amino acid substitution to resistance, the I861T mutation was introduced into JFH1. The sensitivity of the variant to NS2-2 was assessed in the infectious cell culture system. I861T substitution resulted in decrease in NS2-2 potency (Figure 7A). The data suggested that selected I861T substitution within NS2 is the major resistance mutation identified. Although I861T mutation had no effect on viral protein expression (Figure 7B), it escaped the disruption of NS2-2 aptamer on the interaction of NS2 with NS5A (Figure 7C).

**Figure 7:** I861T substitution in NS2 is the major selective resistance mutation identified. (**A**) Selection of resistance-conferring mutations was performed. Huh7.5 cells were infected with media from Huh7.5 cells transfected with RNA from wild type (WT) or selected I861T viral clone. The effect of aptamer NS2-2 on the production of infectious WT or selected I861T mutated virus particles was tested as described in Figure 3D. Results are the average of three independent experiments. *P<0.05, **P<0.01 verse control cells. (**B**) I861T mutation had no effect on viral protein expression. Huh7.5 cells were infected with media from Huh7.5 cells transfected with RNA from wild type (WT) or selected I861T viral clone, followed with NS2-specific aptamer treatment for 72 hours. Protein was isolated and NS2 or NS5A was detected by western blot analysis. (**C**) I861T mutation escaped the disruption of NS2-2 aptamer on the interaction of NS2 with NS5A. Huh7.5 cells were treated as described in part B. Protein was isolated from the HCV-infected Huh7.5 cells with aptamer or library treatment and immunoprecipitated with antibodies against NS5A or mouse IgG conjugated with agarose beads respectively. The protein binding to the beads were boiled and subjected to SDS-PAGE. The protein was transferred onto PVDF membrane and then reacted with mouse monoclonal anti-NS2 or NS5A antibody and secondary antibodies.

## Discussion

Almost half of the individuals infected with HCV genotype 1 do not response to the current pegylated IFN-α-based therapy. The protease inhibitors against NS34A have been recently approved for the treatment of chronic hepatitis C patients [24]. Viral escape mutants resistant to these drugs have already emerged [25]. For an efficient and sustainable therapy against HCV infection, a strategy targeting multiple enzymatic activities or other functions of viral proteins has the best chance for success. Every step of the HCV lifecycle can be a target for novel anti-HCV drugs [26].

NS2 protein is essential for HCV lifecycle, making it an attractive target for antiviral therapies. In the study we selected aptamers against NS2 protein using SELEX and explored the mechanisms of their antiviral effects. To our knowledge, this is the first report of NS2 inhibitors mediating inhibition of HCV infection. We showed that NS2-specific aptamer NS2-2 inhibits virus assembly and release. Moreover, NS2 aptamer inhibits HCV genotype 1a, 1b and 2a infection.

There are relatively few data on the mechanisms of how HCV assemble and release. Several studies showed that NS2 is essential for the production of infectious virus. However, its roles in the HCV lifecycle are still unknown. Although the aptamer NS2-2 was found to bind N-terminal region of NS2 protein (26–93 aa), the detail residues involved in the interaction between NS2-2 aptamer and its target need to be explored. Determination of these residues may provide information about the essential functional regions of NS2. The aptamer NS2-3 was found to bind N-terminal region of NS2 protein. It has been reported that the host proteins interacting with NS2 are essential for HCV RNA replication [27]. The aptamer NS2-3 might indirectly inhibit HCV RNA replication through disrupting the interaction of NS2 with host proteins which are involved in the viral RNA replication. NS2-3 inhibits viral RNA replication and as a result also inhibits virus production. Aptamer against NS2 can be used with NS2 to understand the mechanisms of how HCV replicates and assembles. NS2-specific aptamers provide a powerful tool to explore the interaction between NS2 and host factors. The interaction between the aptamers against HIV reverse transcriptase and reverse transcriptase provides a model for the study of the mechanisms of how these aptamers act as broad-spectrum inhibitors of reverse transcriptase [28]. The aptamers targeting HIV Gag protein can be used to examine the Gag-HIV RNA interactions and can be an effective tool to perturb Gag-genomic RNA interactions [29]. All these examples illustrate the potential use of aptamers in exploring the roles of viral proteins in virus lifecycle and the interaction between virus and host factors. Continue research will aim to elucidate the modes of action of NS2-specific aptamers to further our understanding the functions of NS2 and to develop novel NS2 inhibitors with a higher genetic barrier to resistance.

The fact that intracellular and extracellular infectivity was reduced 50% and 70% respectively by aptamer NS2-2 is consistent with defects in both virus assembly and release. Interaction of NS2 with NS5A protein is critical for infectious HCV production and disruption of this interaction impairs the production of infectious virus. Here we demonstrated that NS2-2 aptamer for NS2 protein disrupts the NS2-NS5A interaction and inhibits infectious virus production.

One recent study reported that inhibition of viral infection by aptamers might be due to the aptamer-induced innate immunity [30]. It is one exceptional example because RIG-I aptamer was designed to have specific motifs to bound and activated RIG-I. Most studies suggest that inhibition of viral infection by aptamers targeting viral proteins attributes to suppression of the functions of viral proteins by aptamers [31]–[34]. In consistent with these studies, our data showed that aptamers against NS2 did not induce IFN-β and ISGs, indicating that inhibition of HCV infection by NS2-specific aptamers is not due to the innate immunity.

In summary, our study provides the first evidence of direct antiviral activity of NS2 aptamers in vitro. These results demonstrate the power of SELEX approach for the selection of inhibitors for viral infection and exploring the mechanisms of viral infection. The data indicate that NS2-2 aptamer for NS2 exerts its antiviral effects through disrupting the interaction of NS2 with NS5A protein. NS2-specific aptamers can be used to understand the mechanisms of virus assembly and release. The aptamers against NS2 may be served as potential drugs for the treatment of chronic hepatitis C patients.
